# A Review on Medicinal Plants Used in the Management of Respiratory Problems in Ethiopia over a Twenty-Year Period (2000–2021)

**DOI:** 10.1155/2022/2935015

**Published:** 2022-06-27

**Authors:** Abebe Ayele Haile, Berhanu Abraha Tsegay, Ali Seid, Wubet Adnew, Admasu Moges

**Affiliations:** ^1^Department of Biology, Bahir Dar University, P.O. Box 79, Bahir Dar, Ethiopia; ^2^Department of Biology, Debre Berhan University, P.O. Box 445, Debre Berhan, Ethiopia

## Abstract

This review is aimed at assessing and compiling the different ethnomedicinal studies in different parts of Ethiopia used to treat respiratory diseases. The data were collected from different published research papers through searching the web sources such as PubMed, Science Direct, Google Scholar, and other related websites. The important search terminologies included ethnobotany, respiratory diseases, medicinal plants, and Ethiopia. For this, a total of 65 articles of recent publications (from 2000 to May 2021 years) that provided full information about the use of medicinal plant species to treat respiratory disorder diseases in Ethiopia were consulted. Based on this, a total of 96 medicinal plants belonging to 57 families were reviewed. The commonly recorded families used to manage respiratory problems were Asteraceae, Lamiaceae, Solanaceae, and Fabaceae. Herbs and shrubs were the dominant plant growth forms. Due to the easiest form of their preparation for treating respiratory disorders, leaves are the most cited plant parts followed by roots. Crushing and pounding are useful methods of remedy preparation to treat respiratory diseases. This review concluded that different medicinal plants have a significant contribution in combating serious respiratory problems in Ethiopia. Hence, the complied review of medicinal plants on the treatment of respiratory problems would play a great role in further pharmacological and phytochemical investigations in developing new drugs used for the treatment of respiratory problems and in the conservation of these important medicinal plants.

## 1. Introduction

The respiratory system is a network of organs and tissues that make respiration possible by making the body absorb oxygen from the air so that organs can function. It cleanses the blood of harmful gases such as carbon dioxide. The respiratory organ system includes airways, the lungs, and blood vessels. The respiratory system can be divided into the upper and lower respiratory tracts. Due to its size, the respiratory system is constantly exposed to microbes [1]. Respiratory infections are the most common of all human infections [2, 3]. This infection is a major cause of death, especially in patients with severe disease. Lower respiratory tract infections have a wide range of symptoms, including acute bronchitis, pneumonia, and chronic obstructive pulmonary disease, which can include symptoms such as cough, nausea, dyspnoea, shortness of breath, and/or chest pain. Common problems include a series of illnesses, including allergies. The incidence and severity of these diseases continue to be high both in developed and developing countries [4]. Upper respiratory tract infections can be defined as self-limited irritation and swelling of the upper airways with associated cough and no signs of pneumonia, in a patient with no other condition that would account for their symptoms, or with no history of chronic obstructive pulmonary disease, emphysema, or chronic bronchitis [5, 6]. Upper respiratory tract infections involve the nose, sinuses, pharynx, larynx, and large airways. The most common respiratory problems are asthma, bronchitis, colds, and coughs [7]. The World Health Organization (WHO) estimates that noncommunicable diseases (NCDs) represent 63% of all global deaths of which 3.9 million are due to chronic respiratory diseases (CRDs) and chronic obstructive pulmonary disease (COPD) in particular [8]. In 2001, noncommunicable diseases accounted for 54% of deaths in low and middle income (developing) countries and 87% of deaths in high income (developed) countries [9]. The global and national burden and threat of noncommunicable diseases (NCDs) constitute a major public health challenge of the 21^st^ century that undermines the social and economic development worldwide and in Ethiopia. To mitigate their impact urgent action is required.

Acute pneumonia is a major cause of infant mortality in the world, accounting for 16% of all deaths worldwide. Some studies have also reported that high rates of acute respiratory infections in Ethiopia range from 16% to 33.5% [10]. In third world countries, where effective air pollution reduction strategies are inadequate, individuals are constantly exposed to substances that have negative health effects in the short and long term [11]. Various vulnerabilities are related to chronic respiratory diseases, including smoking habits, environmental conditions, and personal cooking/heating pollution [12–16].

With regard to the cure of these highly treatable respiratory diseases, the World Health Organization (WHO) is promoting herbal medicine and pharmacological research to make better use of herbal remedies [17]. The use of herbal remedies for the treatment of respiratory disorders is common practice in many parts of the world [18]. Traditional medicine has been an important source of products for developing countries in treating common infections [19].

Medicinal plants are very vital in their uses for medication, besides providing ecological, economic, and cultural services. The world's primary means of treating diseases and fighting infections have been based on the use of medicinal plants. From ancient times, plants have been a rich source of effective and safe medicines [20]. In the world, 64% of the population relies on medicinal plants to treat health problems [21].

In Ethiopia, there are different medicinal plants that are used to treat various respiratory ailments like *Zingiber officinale* Roscoe, *Ocimum lamiifolium* Hochst. ex. Benth, *Artemisia abyssinica* Sch. Bip. ex A. Rich, *Carthamus tinctorius* L, and *Solanecio gigas* (Vatke) C. Jeffrey. However, the effectiveness of these medicinal plants has not yet been scientifically investigated. Recent studies revealed that antimicrobial medicinal plants were investigated scientifically in different countries [22, 23]. Some of the medicinal plants used to treat respiratory disorders were investigated experimentally in vitro such as the extracts from *Gnaphalium oxyphyllum* Steetz ex Griseb, *Gnaphalium americanum* Mill, and *Crescentia alata* Kunth possessed strong antimicrobial activity against *Staphylococcus aureus*, *Enterococcus faecalis*, *Streptococcus pneumoniae*, *Streptococcus pyogenes*, and *Candida albicans* [19]. Moreover, the oils of *Lavandula augustifolia* Mill, *Elettaria cardamomum* (L.) Maton, and *Cymbopogon nardus* (L.) Rendle are major constituents against respiratory tract pathogens by gaseous contact [24]. Kariuki and Njoroge [25] similarly reported that methanolic extracts of *Acacia nilotica* and *Strychnos heninningsii* showed efficacy against *S. aureus, S. pneumoniae,* and *E. coli* [25].

Panax ginseng aqueous extract prevents pneumococcal sepsis in vivo by potentiating cell survival and diminishing inflammation. Taken together, 100 mg/kg of KRG appeared to protect host cells from lethal pneumococcal sepsis by inhibiting inflammation as well as by enhancing bacterial clearance thereby reinforcing cell survival against pneumococcal infection [26].

Ginseng has been traditionally used in Asia for thousands of years to treat a variety of ailments including respiratory diseases. Various studies have shown that both families of compounds can modulate various parameters of the immune response in vitro and in vivo [27]. In clinical trials, healthy subjects that consumed a standardized ginseng extract had a lower incidence of influenza and colds, higher antibody titers, and higher natural killer cell activity [28], as well as increased numbers of total lymphocytes and T helper cells [29]. Ginseng polysaccharide preparations increased cytokine production and mRNA expression by murine macrophages and spleen cells in vitro [30].

The present study is aimed at documenting the traditional uses of medicinal plants used to treat different respiratory disorders in Ethiopia. This review describes the traditional uses of medicinal plants used for the treatment of respiratory disorders in Ethiopia. In general, this review is initiated to identify research gaps and to suggest perspectives for future research in the development of drugs used to treat various respiratory disorders.

## 2. Materials and Methods

### 2.1. Search Strategy

A systematic review of medicinal plants used to treat respiratory disorders in Ethiopia was conducted.

The data for this review were collected from different published articles via downloading them from web sources of PubMed, Science direct, Google scholar, and other related web sites following [31]. Accordingly, ethnobotanical/ethnomedicinal studies reporting on medicinal plants used for traditional respiratory disorder treatment in Ethiopia were gathered through different search approaches such as the Google search engine for published journal articles using international scientific databases including PubMed, Science Direct, Web of Science, and Google scholar. Similarly, missing information from some studies, especially the local, scientific, and family names of plants, was retrieved from the African Natural Database (NDA), version 2.0, as well as online plant scientific checking system for some other plant species was applied. During the search, the terms such as “medicinal plants,” “Ethnobotanical study,” and “Ethiopia or Indigenous people,” “respiratory medicinal plants,” “cough/traditional medicinal plants,” “common cold/traditional medicinal plants,” “nasal bleeding/traditional medicinal plants,” “tonsillitis/traditional medicinal plants,” etc. were used. The medicinal plants used to treat respiratory disorders were included based on the eligibility criteria as described below.

### 2.2. Inclusion and Exclusion Criteria

Articles published only from 2000 to May 2021 were selected. Accordingly, the data collected from the literature included the plant species and its parts, used growth forms, local names, and modes of preparation and/or application. Moreover, the literature search was done to document the biological and pharmacological activities of mostly used plant species for treatment of respiratory disorder problems.

As depicted in Figure 1, 2502 articles were downloaded from different web sources. However, only 65 articles that provided full information about the use of medicinal plant species to treat respiratory disorder diseases in Ethiopia were selected and considered for this review paper (Figure 1).

## 3. Results and Discussion

### 3.1. Composition and Diversity of Medicinal Plants Used to Treat Respiratory Disorders

The reviews made from 65 articles identified 96 medicinal plants that contain full information on how to treat respiratory disorders in the country (Table 1). These plants were collected from different regions. Many of them were collected from Amhara (55.1%), Oromia (23.71%), SNNP (22.45%), and Tigray (6.122%) regional states (Figures 2 and 3), which cover close to 90–95% of the land size of the country, Ethiopia. This is consistent with other reviews made by Megersa et al. [85] on the treatment of toothache and [31] on the treatment of malaria, and also by Bitew et al. [86] on the treatment of wounds. This indicated that other regions were given less attention towards ethnobotanical study, which might be due to their being less studied and having a small land area compared to other regions mentioned here.

According to this review, of the total (96), 16.66% medicinal plants belonged to the Asteraceae and Lamiaceae families, which are equally dominant (Figure 4). Many ethnobotanical studies showed that the family Asteraceae was ranked first at the family level as indicated by Tesfaye et al. [32, 87]. This indicates that many of the medicinal plants used for treating respiratory disorders belong to the two dominant families, and that giving priority to these families in the conservation of medicinal plants is very vital.

### 3.2. Habits (Growth Forms) of Medicinal Plants

Herbs were the dominant plant growth form used to treat respiratory illness according to the current review which accounted for 39 (39.8%) plant species followed by shrubs at 36 (37.11%) (Figure 5). This result is consistent with many publications [12, 32, 52].

### 3.3. Plant Parts Used to Treat Respiratory Diseases

Leaves were the most important plant parts used to prepare medicines which accounted for about 31 plant species, while roots were the next most important part of plants which accounted for about 19 (Figure 6). This is in agreement with findings on other diseases [100–105]. Using the leaves of plants for medicinal preparation has advantages for the survival of the mother plants, whereas using the root parts of the medicinal plants could have threats to these medicinal plants because such practices totally remove the mother trees.

### 3.4. Methods of Preparation of Medicinal Plants Used to Treat Respiratory Diseases

Medicinal plants used to treat respiratory diseases are prepared in a variety of ways. The main methods are pounding and crushing (Figure 7). Fresh preparations are usually preferred by herbalists. This finding is in line with [43–47].

### 3.5. Numbers of Medicinal Plants Used to Treat Respiratory Disease

Current studies show that cough is cured by 45 plants and tonsillitis by 34 plants (Table 2). This implies that cough and tonsillitis could be treated by different medicinal plants, so that the shortage of medicinal plants might not be the problem even during the dry seasons. On the contrary, some respiratory diseases such as sore throat, respiratory tract problems, and chest pain can be cured only by one type of medicinal plant (1.03%). This could be a risk for treating these diseases whenever there is a drought and/or other man-made or natural crisis as the medicinal plants might disappear in such situations. This is consistent with Asadbeigi et al. [106, 107]), Marília et al. [108], and Lawal et al. [109], which implies cough and tonsillitis are treated by different plant species.

## 4. Conclusions and Recommendations

From times in memorial, traditional medicinal plants were being used to treat various ailments including respiratory illnesses. In Ethiopia, 96 medicinal plants are being used to cure respiratory problems. It is necessary that attention should be given to the sustainable use of these plant species and further pharmacological studies should be conducted to extract and use the active medicinal ingredients. This study, we believe, is a gateway for many researchers to give more emphasis on how to extract and develop new drugs to treat respiratory health problems.

## Figures and Tables

**Figure 1:** A diagram showing the selection procedures of the articles for this review.

**Figure 2:** Regional states of Ethiopia, where medicinal plants are found and reviewed.

**Figure 3:** Number of ethnobotanical studies which contain full records of medicinal plants used to treat respiratory diseases in different regions of Ethiopia (*Note*. SNNP = South nation and nationality of people; B. Gumuz = Benishangul Gumuz).

**Figure 4:** Taxonomic diversity of the families of medicinal plants with their percentages in the study area.

**Figure 5:** Growth forms of medicinal plants used to treat respiratory diseases.

**Figure 6:** Plant parts used to treat respiratory diseases.

**Figure 7:** Preparation of medicinal plants used to treat respiratory diseases.

**Table 1:** List of Ethiopian medicinal plants used to treat respiratory diseases. Description of data (Or = afanOromo, Am = Amharic, Tig = Tigrigna, Sd = sidamegna, Daw = dawuro, KA = Kara, KW = Kwego, Ged = Gedeoffa, Kr = Koorete, Ko = konta, Br = Berta).

Plant family	Scientific name	Online references for each plant species	Local name	Habit	parts used	Preparation methods	Traditional use	References
Acanthaceae	*Justicia schimperiana* (Hochst. Ex Nees) T.Anders.	https://www.plantsoftheworldonline.org/taxon/urn:lsid:ipni.org:names:51563-1	Smiza/sensl (Am)	Shrub	Leaf	Rubbing& sniffed	Common cold	[32]
Acanthaceae	Hypoestes forskaolii (Vahl) R.Sch	https://www.plantsoftheworldonline.org/taxon/urn:lsid:ipni.org:names:941349-1	Girbia (Tig)	Herb	Root	Fumigation	Cough	[33, 34]
Alliaceae	*Allium sativum* L	https://www.plantsoftheworldonline.org/taxon/urn:lsid:ipni.org:names:528796-1	Shinkurt (Am)	Herb	Bulb & leaf	Chewed; chopped, pounded	Tonsillitis, cough, common cold	[35, 36]
Amaranthaceae	*Achyranthes aspera* L	https://www.plantsoftheworldonline.org/taxon/urn:lsid:ipni.org:names:2468-2	Telenj (Am)	Herb	Leaf	Crush	Tonsillitis	[32, 37, 38]
Anacardiaceae	*Schinus molle* L.	https://www.plantsoftheworldonline.org/taxon/urn:lsid:ipni.org:names:71044-1	Qudabarbare (oro)	Tree	Seed	Chewed	Tonsillitis	[32, 39]
Annonaceae	*Uvaria leptocladon* Oliv.	https://www.plantsoftheworldonline.org/taxon/urn:lsid:ipni.org:names:75780-1	Zebko (KA) Chochum (kw)	Tree	Root	Crushed/decoction/boiled	Cough, chest pain	[40]
Apiaceae	*Foeniculum vulgare* Miller	https://www.plantsoftheworldonline.org/taxon/urn:lsid:ipni.org:names:842680-1	Ensilal (Am)	Herb	Above ground	Boiled	Cough	[32, 41]
Apiaceae	*Coriandrum sativum* L.	https://www.plantsoftheworldonline.org/taxon/urn:lsid:ipni.org:names:840760-1	Dimbilal (Am)	Herb	Seed	Grounded	Cough	[42]
Apiaceae	*Nigella sativa* L.	https://www.plantsoftheworldonline.org/taxon/urn:lsid:ipni.org:names:711687-1	Tiqur-azmud (Am)	Herb	Seed	Grounded	Common cold Asthma	[43, 44]
Apocynaceae	*Carissa spinarum* L	https://www.plantsoftheworldonline.org/taxon/urn:lsid:ipni.org:names:77756-1	Laadiya (daw) Otilaa (Sd)	Shrub	Leaf& fruit	Chewed; Chopped, Ground	Tonsillitis	[35, 45, 46]
Asclepiadaceae	*Kanahia laniflora* (Forssk.) R.Br	https://www.plantsoftheworldonline.org/taxon/urn:lsid:ipni.org:names:98887-1	Tifrindo (Am.) Wundiffo (Ged)	Herb	Root/leaf	Sniffing, inhaling	Flue, asthma bronchitis	[47, 48]
Asparagaceae	*Asparagus africanus* Lam	https://www.plantsoftheworldonline.org/taxon/urn:lsid:ipni.org:names:530996-1	Yeset kest (Am)	Herb	Root	Boiled, decoction	Cough	[49]
Asteraceae	*Echinops kebericho* Mesfin	https://www.plantsoftheworldonline.org/taxon/urn:lsid:ipni.org:names:940177-1	Kebericho (Am)	Herb	Bulb	Smoked	Cough	[50]
Asteraceae	*Acmella caulirhiza* Del	https://www.plantsoftheworldonline.org/taxon/urn:lsid:ipni.org:names:174533-1	Gutichaa (Oro)	Herb	Flower	Chewed and spitted	Tonsillitis	[51, 52]
Asteraceae	*Laggera tomentosa* (Sch. Bip.ex A. Rich.) Oliv. & Hiern	https://www.plantsoftheworldonline.org/taxon/urn:lsid:ipni.org:names:60455903-2	Nech kese (Am)	Herb	Leaf	Holding	Common cold/cough	[53]
Asteraceae	*Vernonia amygdalina* Delile	https://www.plantsoftheworldonline.org/taxon/urn:lsid:ipni.org:names:257798-1	Grawa (Am)	Shrub	Leaf	Crushed	Tonsillitis	[54]
Asteraceae	*Kleinia abyssinica* (A. Rich.) A. Berger	https://www.plantsoftheworldonline.org/taxon/urn:lsid:ipni.org:names:227346-1	Este-maza (Am)	Herb	Leaf	Squeezed, drunk	Tonsillitis	[55]
Asteraceae	*Helianthus annuus* L	https://www.plantsoftheworldonline.org/taxon/urn:lsid:ipni.org:names:119003-2	Suf (Am)	Herb	Seed	Decoction	Coughing, common cold	[56]
Asteraceae	*Artemisia absinthium* L	https://www.plantsoftheworldonline.org/taxon/urn:lsid:ipni.org:names:300106-2	Aritii (oro) (Am)	Herb	Root & leaf	Pounded	Sour throat/tonsillitis	[51, 57]
Asteraceae	*Guizotia abyssinica* (L.f.) Cass.	https://www.plantsoftheworldonline.org/taxon/urn:lsid:ipni.org:names:210735-1	Nug (Am)	Herb	Seed	Pounded	Dry cough	[58]
Balsaminaceae	*Impatiens ethiopica* Grey-Wilson	https://www.plantsoftheworldonline.org/taxon/urn:lsid:ipni.org:names:103607-1	Insosla (Am)	Herb	Root	Crushing and Pounding	Cough	[59]
Boraginaceae	*Trichodesma zeylanicum (Burm. f.) R. Br*	https://www.plantsoftheworldonline.org/taxon/urn:lsid:ipni.org:names:121302-1	Jgewusha (Gum)	Shrub	Root	Crushed, squeezed	Tonsillitis	[60]
Brassicaceae	*Lepidium sativum* L.	https://www.plantsoftheworldonline.org/taxon/urn:lsid:ipni.org:names:138141-2	Feecoo (oro)/feto (Am)	Herb	Seed	Pounded	Cough & tonsillitis	[39]
Brassicaceae	*Brassica nigra* (L) Czern	https://www.plantsoftheworldonline.org/taxon/urn:lsid:ipni.org:names:60442520-2	Sanafica (oro)	Herb	Seed	Pounded	Common cold	[61]
Canellaceae	*Warburgia ugandensis* Sprague	https://www.plantsoftheworldonline.org/taxon/urn:lsid:ipni.org:names:146038-1	Beft (oro)	Tree	Stem	Sniffed smoke	Cough	[62]
Capparidaceae	*Capparis tomentosa* Lam.	https://www.plantsoftheworldonline.org/taxon/urn:lsid:ipni.org:names:146824-1	Gumero (Am)	Shrub	Root, fruit	Grinding, chewing	Tonsillitis	[43]
Caricaceae	*Carica papaya* L.	https://www.plantsoftheworldonline.org/taxon/urn:lsid:ipni.org:names:77126657-1	Papaya (Am)	Tree	Root	Crushed and boiled	Cough	[32]
Celastraceae	*Catha edulis* (Vahl) Endl	https://www.plantsoftheworldonline.org/taxon/urn:lsid:ipni.org:names:941530-1	Chat (Am)	Shrub	Leaf & stem	Boiled, drunk	Cough	[63]
Crassulaceae	*Kalanchoe laciniata* (L) DC	https://www.plantsoftheworldonline.org/taxon/urn:lsid:ipni.org:names:274383-1	Anchura (oro)	Herb	Root	Pounded	Cough	[64]
Cucurbitaceae	*Momordica foetida* Schumach	https://www.plantsoftheworldonline.org/taxon/urn:lsid:ipni.org:names:293451-1	Yubarrae (Ged) Yekurahareg (Am) Suruphaa (oro)	Shrub	Roots	Crushed pounded	Bronchitis tonsillitis	[32, 47]
Cucurbitaceae	*Cucumis ficifolius* A. Rich	https://www.plantsoftheworldonline.org/taxon/urn:lsid:ipni.org:names:292191-1	Yemidir Embuy (Am)	Climber	Root	Washed, smashed mixed with water	Cough bronchitis	[43, 65]
Cupressaceae	*Juniperus procera* Hochst. ex Endl.	https://www.plantsoftheworldonline.org/taxon/urn:lsid:ipni.org:names:262311-1	Yehabeshatsid (Am)	Herb	Stem/root	Grinding/boiling	Cough	[62]
Euphorbiaceae	*Euphorbia schizacantha* Pax	https://www.plantsoftheworldonline.org/taxon/urn:lsid:ipni.org:names:348181-1	Dhetungayda (Kr)	Herb	Leaf	Pounded	Cough	[50]
Euphorbiaceae	*Tragia pungens* (Forssk.) Muell. Arg	https://www.plantsoftheworldonline.org/taxon/urn:lsid:ipni.org:names:357857-1	Aleblabit (Am)	Climber	Root & leaf	Powdered, boiled decoction	Chronic cough (T.B)	[66]
Euphorbiaceae	*Croton macrostachyus* Hochst. ex Delile	https://www.plantsoftheworldonline.org/taxon/urn:lsid:ipni.org:names:342917-1	Mesana (Oro) Bisana (Am)	Tree	Twig	Crushed, drunk	Tonsillitis Asthma	[60, 67]
Euphorbiaceae	*Ricinus communis* L	https://www.plantsoftheworldonline.org/taxon/urn:lsid:ipni.org:names:355498-1	Qolompo desha (kw) Ati (ka, kw)	Tree	Root	Chewing/crushed boiled	Flu	[40, 68]
Fabaceae	*Albizia amara* (Roxb.) Boivin	https://www.plantsoftheworldonline.org/taxon/urn:lsid:ipni.org:names:473171-1	Ondoddee (Kr)	Tree	Leaf	Crushed	Cough	[48, 53]
Fabaceae	*Acacia tortilis* (Forssk.) Hayne	https://www.plantsoftheworldonline.org/taxon/urn:lsid:ipni.org:names:471662-1	Tadacha (Am)	Tree	Leaf	Concoction	Throat infection	[69]
Fabaceae	*Acacia nilotica* (L.) P.J.H.Hurter & Mabb.	https://www.plantsoftheworldonline.org/taxon/urn:lsid:ipni.org:names:77089275-1	Kasalto [Af]	Tree	Stem bark	Infusion	Tonsillitis	[70]
Fabaceae	*Tephrosia elata* Deflers	https://www.plantsoftheworldonline.org/taxon/urn:lsid:ipni.org:names:520536-1	Kashabach (Tig)	Shrub	Root	Grounded	Respiratory tract problem	[71]
Fabaceae	*Acacia oerfota* (Forssk.) Schweinf	https://www.plantsoftheworldonline.org/taxon/urn:lsid:ipni.org:names:520536-1	Ajo (oro)	Shrub	Bark	Chewed	Tonsillitis	[72]
Flacourtiaceae	*Dovyalis abyssinica* (A. Rich.) Warb.	https://www.plantsoftheworldonline.org/taxon/urn:lsid:ipni.org:names:111558-1	Koshim (Am)	Shrub	Leaf	Boiling	asthma	[58]
Lamiaceae	*Ocimum lamiifolium* Hochst. Ex Benth.	https://www.plantsoftheworldonline.org/taxon/urn:lsid:ipni.org:names:453009-1	Damakase (Ged) (Am)	Herb	Leaf	Pounded	Cough/nose bleeding/Influenza	[47, 73]
Lamiaceae	*Clerodendrum myricoides* (Hochst.) R.Br. Ex Vatke	https://www.plantsoftheworldonline.org/taxon/urn:lsid:ipni.org:names:862273-1	Misrich (Am)/ Bishchereh (Br)	Shrub	Root bark	Decocted	Dry cough/common cold	[64, 74]
Lamiaceae	Thymus serrulatus Hochst. ex Benth.	https://www.plantsoftheworldonline.org/taxon/urn:lsid:ipni.org:names:461653-1	Tosigne (Am)	Herb	Leaf	Boiled	Whooping cough	[73, 75]
Lamiaceae	*Clerodendrum* alatum Gurke	https://www.plantsoftheworldonline.org/taxon/urn:lsid:ipni.org:names:861906-1	Misirich (Am)	Herb	Bark	Pounded	Tonsillitis	[37]
Lamiaceae	Ajuga integrifolia Buch.-Ham. ex D.Don	https://www.plantsoftheworldonline.org/taxon/urn:lsid:ipni.org:names:444595-1	Tut astil (Am)	Herb	Leaf	Rubbed, Squeezed	Tonsillitis	[54]
Lamiaceae	*Mentha spicata* L	https://www.plantsoftheworldonline.org/taxon/urn:lsid:ipni.org:names:30016176-2	Nana (oro)	Herb	Leaf	Boiled, drunk	Cough and cold	[57]
Lamiaceae	*Ranunculus multifidus* Pursh	https://www.plantsoftheworldonline.org/taxon/urn:lsid:ipni.org:names:217450-2	Afi Deshe (Am)	Herb	Leaf	Pounded	Tonsillitis	[76]
Lamiaceae	*Otostegia fruticosa* (Forssk.) Schweinf. Ex penzig	https://www.plantsoftheworldonline.org/taxon/urn:lsid:ipni.org:names:453638-1	Tunjut (Am)	Shrub	Leaf	Burning	Common cold	[77]
Loganiaceae	*Buddleja polystachya* Fresen.	https://www.plantsoftheworldonline.org/taxon/urn:lsid:ipni.org:names:545859-1	Anfar (Am)	Shrub	Shoot	Concoction	Tonsillitis	[32, 78]
Loganiaceae	*Nuxia congesta* R.Br. Ex Fresen.	https://www.plantsoftheworldonline.org/taxon/urn:lsid:ipni.org:names:546816-1	Atquar (Am)	Shrub	Shoot	Rub, squeeze	Tonsillitis	[32]
Malvaceae	*Gossypium barbadense* L.	https://www.plantsoftheworldonline.org/taxon/urn:lsid:ipni.org:names:559677-1	Tit (Am)	Shrub	Fruit	Grinded	Tonsillitis	[32]
Malvaceae	*Sida rhombifolia* L	https://www.plantsoftheworldonline.org/taxon/urn:lsid:ipni.org:names:235798-2	Karaba (Oro)	Shrub	Leaf	Boiled	Asthma	[79]
Meliaceae	*Azadirachta indica* A. Juss.	https://www.plantsoftheworldonline.org/taxon/urn:lsid:ipni.org:names:1213180-2	Nim (Am)	Tree	Leaf	Boiled	Cough	[59]
Meliantaceae	*Bersama abyssinica* Fresen	https://www.plantsoftheworldonline.org/taxon/urn:lsid:ipni.org:names:782127-1	Xibiro (oro)	Shrub	Root	Crushed	Bronchitis	[61, 69]
Menispermaceae	Stephania abyssinica (Quart.-Dill. & A.Rich.) Walp	https://www.plantsoftheworldonline.org/taxon/urn:lsid:ipni.org:names:581384-1	Chewchawit (Am)	Herb	Shoot	Crushed	Tonsillitis	[32]
Moraceae	*Dorstenia barnimiana* Schweinf	https://www.plantsoftheworldonline.org/taxon/urn:lsid:ipni.org:names:60453283-2	Work Bemeda (Am)	Herb	Root	Infusion	Acute coughing	[79]
Myrataceae	*Eucalyptus globulosus* St.-Lag	https://www.plantsoftheworldonline.org/taxon/urn:lsid:ipni.org:names:592964-1	Tsaedakelamitos (Tig)	Tree	Leaf	—	Cough	[80]
Myricaceae	*Myrica salicifolia* Hochst. ex A.Rich.	https://www.plantsoftheworldonline.org/taxon/urn:lsid:ipni.org:names:585605-1	Shinet (Am)	Tree	Bark	Crushed, powdered	Common cold & bleeding	[32]
Myrsinaceae	*Maesa lanceolata* Forssk	https://www.plantsoftheworldonline.org/taxon/urn:lsid:ipni.org:names:588843-1	Geggec'uwa (daw)	Tree	Leaf, bark and seed	Chopped, Pound; ground	Tonsillitis	[35]
Myrtaceae	Syzygium guineense (Willd.) DC.	https://www.plantsoftheworldonline.org/taxon/urn:lsid:ipni.org:names:601750-1	Ochaa (daw)	Tree	Leaf root and bark	Chopped	Tonsillitis/flu & sore throat	[35]
Myrtaceae	*Eucalyptus globulus* Labill.	https://www.plantsoftheworldonline.org/taxon/urn:lsid:ipni.org:names:592965-1	Nech bahrzaf (Am)	Tree	Leaf	Burning	Common cold	[36]
Nyctaginaceae	*Commicarpus sinuatus* Meikle	https://www.plantsoftheworldonline.org/taxon/urn:lsid:ipni.org:names:604483-1	Kontom (Or)	Herb	Leaf	Concoction	Throat infection	[69]
Olacaceae	*Ximenia americana* L	https://www.plantsoftheworldonline.org/taxon/urn:lsid:ipni.org:names:316341-2	Hudhaa (oro) Mekela (KA) Waljoweljo (KW)	Shrub	Root	Crushed, pounded	Tonsillitis, Flu	[40, 57]
Oleaceae L.	*Olea europaea*	https://www.plantsoftheworldonline.org/taxon/urn:lsid:ipni.org:names:610675-1	Woira (Am)	Tree	Leaf	Chewed	Tonsillitis	[32]
Phytolaccaceae	*Phytolacca dodecandra* L'Her	https://www.plantsoftheworldonline.org/taxon/urn:lsid:ipni.org:names:676349-1	Shebti (Tig)	Shrub	Root	Juice	Cough	[81]
Piperaceae	*Piper capense* L.f.	https://www.plantsoftheworldonline.org/taxon/urn:lsid:ipni.org:names:680780-1	Timiz (Am)	Shrub	Seed	Powdered	Cold, cough	[56]
Plumbaginaceae	*Plumbago zeylanica* L	https://www.plantsoftheworldonline.org/taxon/urn:lsid:ipni.org:names:687109-1	Amira (Am)	Shrub	Leaf	Boiled, drunk	Cough asthma	[82]
Poaceae	*Cymbopogon citratus* (DC.) Stapf	https://www.plantsoftheworldonline.org/taxon/urn:lsid:ipni.org:names:396896-1	Xajisaara (oro)	Herb	Leaf	Burnt	Cough	[57]
Poaceae	*Saccharum officinarum* L.	https://www.plantsoftheworldonline.org/taxon/urn:lsid:ipni.org:names:419977-1	Shankora (Am)	Shrub	Stem	Ate	Common cold	[83, 84]
Podocarpaceae	Podocarpus gracilior Pilg.	https://www.plantsoftheworldonline.org/taxon/urn:lsid:ipni.org:names:263490-1	Zigba (Am)	Tree	Sap	Crushing	Common cold	[28–89]
Polygalaceae	Polygala obtusissima Hochst. ex Chodat	https://www.plantsoftheworldonline.org/taxon/urn:lsid:ipni.org:names:691954-1	Calmala [Af]	Shrub	Leaf	Pounded	Common Cold	[69]
Polygonaceae	*Rumex nepalensis* Spreng	https://www.plantsoftheworldonline.org/taxon/urn:lsid:ipni.org:names:697338-1	Zans'alaa (dawro)/tult (Am) Tultii (oro)	Herb	Root &leaf	Chewed	Tonsillitis	[35, 90]
Ranunculaceae	Clematis hirsuta Guill. & Perr.	https://www.plantsoftheworldonline.org/taxon/urn:lsid:ipni.org:names:709771-1	Azo Hareg (Am)	Climber	Leaf	Juice	Cough	[91]
Rhamnaceae	*Rhamnus prinoides* L'Herit	https://www.plantsoftheworldonline.org/taxon/urn:lsid:ipni.org:names:718580-1	Geeshuwa (daw) Geeshoo (oro)	Shrub	Leaf	Pounded; Chewed	Tonsillitis	[35, 92]
Rosaceae	*Prunus Africana* (Hook.f) Kalkman	https://www.plantsoftheworldonline.org/taxon/urn:lsid:ipni.org:names:729417-1	Tikur Inchet (Am)	Tree	Leaf	Pounded	Tonsillitis	[66]
Rubiaceae	*Rubia cordifolia* L	https://www.plantsoftheworldonline.org/taxon/urn:lsid:ipni.org:names:765218-1	Enchibir (Am)	Herb	Root & leaf	Powdered, boiled decoctio,	Cold, cough	[66]
Rubiaceae	*Coffea arabica* L	https://www.plantsoftheworldonline.org/taxon/urn:lsid:ipni.org:names:747038-1	Buna (Am)	Shrub	Seed	Decoction	Asthma	[54]
Rutaceae	Citrus limon (L.) Osbeck	https://www.plantsoftheworldonline.org/taxon/urn:lsid:ipni.org:names:60454758-2	Lomae (Ged) lomi (Am)	Shrub	Fruit	Chew	Cough	[47, 93]
Rutaceae	*Citrus aurantiifolia* (Christm.) Swingle	https://www.plantsoftheworldonline.org/taxon/urn:lsid:ipni.org:names:59599-2	Tutto (kr)	Shrub	Fruit	Juice	Cough	[48]
Rutaceae	*Ruta chalepensis* L.	https://www.plantsoftheworldonline.org/taxon/urn:lsid:ipni.org:names:775070-1	Chelatama (oro)	Shrub	Fruit	Boiled	Cough	[62]
Santalaceae	Osyris lanceolata Hochst. & Steud.	https://www.plantsoftheworldonline.org/taxon/urn:lsid:ipni.org:names:780506-1	Waatoo (oro)	Shrub	Root, stem	Grinding, Powdering	Common cold	[94]
Scrophulariaceae	*Verbascum sinaiticum* Benth	https://www.plantsoftheworldonline.org/taxon/urn:lsid:ipni.org:names:770131-1	Tirnake (Tig)	Herb	Root	Crushed	Tonsillitis	[95]
Solanaceae	*Solanum incanum* L.	https://www.plantsoftheworldonline.org/taxon/urn:lsid:ipni.org:names:819567-1	Hiddi (oro)	Shrub	Fruit	Juice	Tonsillitis	[39]
Solanaceae	*Solanum marginatum* L.f	https://www.plantsoftheworldonline.org/taxon/urn:lsid:ipni.org:names:819994-1	Yedega enboy (Am)	Shrub	Fruit	Juice	Cough	[32]
Solanaceae	*Withania somnifera* (L.) Dunal	https://www.plantsoftheworldonline.org/taxon/urn:lsid:ipni.org:names:821709-1	Giziewa (Am)	Shrub	Leaf	Crushed	Cough/Asthma	[32]
Solanaceae	*Datura stramonium* L	https://www.plantsoftheworldonline.org/taxon/urn:lsid:ipni.org:names:314738-2	Manjii (oro)	Herb	Leaf	Pounded, drunk	Cough	[92]
Solanaceae	*Solanum dasyphyllum* Schumach &Thonn	https://www.plantsoftheworldonline.org/taxon/urn:lsid:ipni.org:names:818913-1	Geber enbuay (Am)	Shrub	Leaf	Crushed	Nosebleed	[96, 97]
Solanaceae	*Solanum incanum* L.	https://www.plantsoftheworldonline.org/taxon/urn:lsid:ipni.org:names:819567-1	Buluwaa (ko)	Shrub	Fruit	Homogenized	Cough	[98]
Tiliaceae	*Grewia ferruginea* Hochst ex A. Rich	https://www.plantsoftheworldonline.org/taxon/urn:lsid:ipni.org:names:834226-1	Ogomdii (Ged)	Shrub	Root bark	Crushed	Cough	[43]
Verbenaceae	*Lippia adoensis* Hochst. ex Walp	https://www.plantsoftheworldonline.org/taxon/urn:lsid:ipni.org:names:863500-1	Kusaayee (oro)	Shrub	Leaf	Pounded, drunk	Cough	[92]
Verbenaceae	*Verbena officinalis* L.	https://www.plantsoftheworldonline.org/taxon/urn:lsid:ipni.org:names:330554-2	Atuch (Am)	Herb	Twig	Crushed	Tonsillitis	[32, 71]
Verbenaceae	*Aloysia triphylla* Britton	https://www.plantsoftheworldonline.org/taxon/urn:lsid:ipni.org:names:9688-2	Xuxxoo (oro)	Tree	Leaf	Pounded	Tonsillitis	[65]
Vitaceae	Cyphostemma adenocaule (Steud. Ex A.Rich.) Desc. ex wild & R.B.Drumm	https://www.plantsoftheworldonline.org/taxon/urn:lsid:ipni.org:names:870171-1	Mrkuszibei (Tig)	Herb	Root	Chewed	Tonsillitis	[53]
Zingiberaceae	Zingiber officinale Roscoe	https://www.plantsoftheworldonline.org/taxon/urn:lsid:ipni.org:names:798372-1	Zinjibilaa (oro) zinjble (Am.)	Herb	Root	Crushed & boiled	Cough, cold& tonsillitis	[54, 64, 99]

**Table 2:** Number of medicinal plants used to treat each type of respiratory diseases.

No	Respiratory disease	Number of medicinal plants	Percentage
1.	Cough	45	46.4
2.	Tonsillitis	34	35.05
3.	Bronchitis	4	4.1
4.	Common cold	16	16.5
5.	Flu	4	4.1
6.	Sore throat	1	1.03
7.	Bleeding	2	2.06
8.	Influenza	1	1.03
9.	Asthma	8	8.25
10.	Respiratory tract problem	1	1.03
11.	Throat infection	2	2.06
12.	Chest pain	1	1.03
